RETRACTED

# Knowledge Discovery-Based Analysis of Health Factors of Urinary Infections in Elderly Cardiology Inpatients

**DOI:** 10.1155/2022/7037037

**Published:** 2022-04-21

**Authors:** Min Zhao, Yan Pi, Longbo Zhang

**Affiliations:** ^1^Department of Cardiovascular Medicine, Chongqing Seventh People's Hospital, Chongqing 401320, China; ^2^Department of Endocrinology and Nephrology, Chongqing Seventh People's Hospital, Chongqing 401320, China; ^3^Urology Surgery, People's Hospital Affiliated to Chongqing Three Gorges Medical College, Wanzhou, Chongqing 404000, China

## Abstract

A set of semantic similarity calculation methods combining full-text text and domain knowledge topics is proposed for the current study of entity association relations such as disease–gene in medical texts combined with topics in knowledge discovery, which is insufficient to reveal the deep semantic association relations of medical domain knowledge at topic level. Taking urinary infections in elderly inpatients as the research subject, word embedding representation of word vectors and topic vectors is performed by the TWE model, and similarity calculation is performed by combining text and domain knowledge topics based on Siamese Network framework. The urinary microbiological culture results of both groups were dominated by *Escherichia coli*, accounting for 34.65% and 47.92%, respectively; the use of antimicrobial drugs in the symptomatic urinary infection group was 94.19% higher than that in the asymptomatic bacteriuria group, 77.27% (*x*^2^  = 8.158, *P*=0.004).

## 1. Introduction

Urinary tract infection (UTI) is an inflammatory response produced by the urinary epithelium after pathogens have invaded the urinary system, usually accompanied by bacteriuria and pyuria. The infection is classified according to the site of infection, and there are different sites of infection such as the kidney, the ureter, the bladder, and the urethra [1].

Depending on the presence or absence of clinical symptoms of infection, there are symptomatic urinary infections and asymptomatic urinary infections (also known as asymptomatic bacteriuria). Urinary infections are common infectious diseases, accounting for the second most common infections in the community and one of the most important hospital infections [2], and urinary tract infections account for about 20.8% to 31.7% of nosocomial infections in China [3]; urinary tract infections in the elderly account for the fourth most common hospital infections in the elderly [4]. Urinary tract infections leading to shock or even death are the 3rd most common among all patients who die from infections [5]. The incidence of urinary infections in elderly patients is high, and studies have shown that urinary infections account for 25% of all elderly patients with infections [6], followed by atypical symptoms, diagnosis, and treatment in the clinic being difficult; acute urinary infections, if not treated in a timely manner, can easily delay the disease and transform into chronic urinary infections, and even cause substantial renal injury and renal failure. Positive urine microbiological culture is the main indicator for the diagnosis of urinary infections, but not all positive cultures require anti-infective treatment, and most patients with asymptomatic bacteriuria do not require anti-infective treatment. The correct distinction between symptomatic urinary infections and asymptomatic bacteriuria is the basis for the rational use of antibacterial drugs. Most past studies on urinary infections in elderly patients in China [7] focused on the factors related to the development of symptomatic urinary infections and the distribution of pathogenic bacteria, while the distribution of pathogenic bacteria between asymptomatic bacteriuria and symptomatic urinary infections was not categorized and analyzed, with the use of antimicrobial drugs and the differential treatments between them being rare [8].

RETRACTED

Cardiology inpatients are generally associated with cardiac insufficiency, reduced cardiac ejection, decreased organ function, and inadequate blood supply to tissues and organs, which, combined with long duration of illness, poor body immunity, and combined underlying diseases, make them highly susceptible to nosocomial infections [9]. At the same time, the immune function and defense mechanisms of elderly cardiology inpatients are decreasing with age, making them a high-risk group for nosocomial infections [10]. In the study, 102 (8.36%) of 1,220 elderly cardiology inpatients developed nosocomial infections, including 70.59% respiratory infections and 29.41% urinary tract infections, which is similar to some reported results [11]. Once infections occur in elderly cardiology patients, it not only increases their physical and mental suffering, but also causes unnecessary waste of medical resources [12]. Therefore, it is imperative to analyze the high-risk factors of nosocomial infections in elderly cardiology inpatients and explore effective intervention programs.

The article found that university and multivariate logistic regression analysis showed that cardiac function grade III-IV, use of ≥2 antimicrobial drugs, use of antimicrobial drugs for ≥2 weeks, length of stay for ≥2 weeks, invasive operations, and other cucurbit diseases were independent risk factors for nosocomial infections in elderly cardiology inpatients, with statistically significant differences (*P* < 0.05) [13]. The higher the cardiac function grade, the more severe the patient's condition; the presence of poor mobility, inadequate tissue blood supply, long hospital stay, and complex treatment protocols can trigger nosocomial infections. The use of many types of antimicrobial drugs for a long time can increase the resistance of drug-resistant strains and add drug-resistant strains, interfering with the balance of the normal flora and causing various pathogenic infections, resulting in nosocomial infections [14, 15].

RETRACTED

The study of medical text similarity computation focuses on obtaining the similarity between sentences by computing word-level similarity, which is then used for knowledge discovery in the medical domain. Currently, there are three main types of medical text similarity computation methods, such as similarity computation based on Gene Ontology GO (Gene Ontology) [9], similarity computation based on topic level [16], and similarity computation based on MeSH word list [17], and other main methods. Among them, [18] demonstrated that a distributed representation based on unsupervised learning of sentences from a large biomedical corpus is not necessarily optimal for domain-specific semantic sentence-level similarity computation, and proposed a method for sentence semantic similarity computation incorporating biomedical ontology. To reduce the burden on clinical researchers and provide decision support, [19] developed an automated text mining method and tool (CHAT), which classifies sentences in the literature based on cancer markers and by calculating the similarity between them it can finally organize and classify cancer-related literature. [20] manually annotated PubMed literature abstracts using MeSH terms and calculated potential associations between terms through co-occurrence relationships between terms and potential associations between MeSH. The method based on word lists and gene ontology in the above study poses some difficulties for the implementation of this method because of the need for pre-tagged corpus and lexical entries. In contrast, there are various methods to obtain literature topics with good extensibility and generalizability.

Therefore, in this study, a deep learning representation was used to explore the similarity computation at the topic level for cardiology inpatients. In order to better learn the information such as words and topics, the semantic information of medical literature at the topic level is learned by the Topic Word Embedding representation model [2] (Topic Word Embedding, TWE), and then the twin neural network model (Siamese Network) [3] in deep learning is used for similarity calculation; the similarity calculation results are used for knowledge discovery analysis based on clustering results.

RETRACTED

## 2. Related Work

Deep learning word embedding representation method represents words as vectors with specific semantic information, and deeper semantic association information can be obtained by similarity calculation. Based on the deep learning medical literature similarity calculation, [13] proposed a new ontology vector representation method OPA2Vec, which combines the ontology and ontology annotation data in PubMed abstracts and obtains the vector representation of ontology by Word2Vec model training, which is finally used for the prediction of protein interaction relationships. [14] Based on the representation of the medical literature abstracts into semantic triads, adversarial networks were used to generate threshold criteria for distinguishing similar texts from more divergent texts, and the effectiveness of the method in information retrieval applications of literature in the clinical domain was demonstrated experimentally. [15] proposed a method for word similarity computation based on deep learning semantic representation using subwords and MeSH word lists, and achieved better results in both sentence similarity computation and biomedical relationship extraction tasks. The above deep learning semantic representation for similarity exploration in the medical domain basically uses only abstract-related information from the literature; however, the study of [1] showed that incomplete gene and disease association relationships included in the abstract may affect the accuracy of the results. Meanwhile, the study of [17] demonstrated that the extraction and automatic classification performance of side effect information of anticancer drugs in medical literature can be effectively improved using the results of drug side effect markers in full-text medical texts. In addition, few investigations have applied the deep learning models that can combine text and topics proposed by [19] and others to the medical field. [20] showed in their study that word embedding models trained in medical collections do not capture well the connections between some specific words, such as heart and related words mentioned in prescriptions, while adding knowledge information to word embeddings can be better applied to medical text representation computational tasks.

## 3. Model Construction

### 3.1. Siamese Network Model-Based Medical Full-Text Similarity Calculation

The Siamese Network model-based medical full-text similarity calculation is divided into the following three parts: (i) text annotation and extraction based on domain knowledge; (ii) similarity calculation based on the Bi LSTM Siamese Network; (iii) text clustering and target gene knowledge discovery. The specific research framework is shown in Figure 1.

RETRACTED

### 3.2. Research Methodology and Steps

#### 3.2.1. Domain Knowledge-Based Text Annotation and Extraction

In this study, the full text of the oncology literature was used for annotation, and the study of [4] showed that the annotation of domain knowledge such as genes and drugs in medical literature abstracts can effectively improve the prediction results of drug indications and side effects. We refer to the annotation system for medical literature in the work of [4], and combined with the actual situation of markup accessibility of the medical full text selected for analysis, a total of disease, gene, causative factor, and drug information was selected for markup. The need for tagging of words appearing in academic full-text texts was mainly based on the word lists in medical databases [7] or on the normative descriptions obtained in the relevant literature. Subsequently, information on diseases, genes, causative factors, and drugs in urinary infections in elderly hospitalized patients was manually labeled according to the labeling rules in the literature [8]. The annotation staff consisted of experts and graduate students in intelligence and medicine. To ensure the quality of the annotation results, manual verification was performed on a case-by-case basis for annotation inconsistencies on the basis of double annotation. Thus, “Ki67,” “expression,” and “breast cancer” were annotated. The number of each medical entity labeled and the statistics of the number of genes labeled in the article are shown in Figures 2 and 3, respectively.

#### 3.2.2. Similarity Calculation Based on the Bi LSTM Siamese Network

*(1) TWE subject word embedding representation*. First, the extraction of relevant topics in full-text journal texts is performed based on the LDA model, and the optimal number of topics is obtained by calculating the perplexity. The LDA model has been shown to be effective for extracting and analyzing topics in the medical field. Subsequently, we perform the word embedding representation of the word–topic pairs generated by the LDA model using the topic word embedding representation, TWE, model, which learns different word embedding representation results for each word under different topics. The specific framework is shown in Figure 4

The TWE model learns topic vector *T*_*i*_ and word vector *W*_*i*_, respectively, using word–topic pairs 〈*W*_*i*_, *T*_*i*_〉 trained in LDA as input, treating each topic as a pseudoWord, and incorporating the topic into the basic word embedding representation by considering that the resulting topic word embeddings acquire different meanings of a word in different contexts. The optimization function of the learning objective of TWE is shown in equation (1):

(1) $$\begin{array}{c} L\left(D\right)=\frac{1}{M}\sum_{i=0}^{M}\sum_{-k,c,k,c\neq 0}\log\;\mathrm{Pr}\left(W_{i+c}|W_{i}\right)+\log\;\mathrm{Pr}\left(W_{i+c}|T_{i}\right). \end{array}$$

In this study, we take the text results of the word–topic distribution generated from urinary infections in elderly inpatients as input and generate word embedding vectors and topic vectors under each tumor topic by training with the TWE model.

*(2) Introduction of the Bi LSTM Siamese Network Model*. The Siamese Network framework is a neural network framework for evaluating the similarity of two input samples, and the framework of the Siamese Network in this study is shown in Figure 5.

RETRACTED

The Siamese Network has two sub-networks with the same structure and shared weights *W*, which receive two input texts D1 and D2 and the label *y* between D1 and D2 in this paper, respectively. This network can better achieve the effective mining of syntactic or semantic association knowledge of two words. The LSTM is composed of four important elements: memory unit *c*_*t*_, input gate *i*_*t*_, output gate *o*_*t*_, and forgetting gate *f*_*t*_. The memory unit *c*_*t*_ determines the memory state based on the current input, the output gate *o*_*t*_ determines how much *c*_*t*_ should be exposed to the next node, and the input gate *i*_*t*_ controls the current input information *w*_*t*_. The forgetting gate *f*_*t*_ determines whether the state information of the previous memory unit should be forgotten. The specific calculation is shown by equations (2) to (7).

(2) $$\begin{array}{c} f_{t}=\sigma \left(U_{f}\left[h_{t-1},w_{t}\right]+b_{f}\right), \end{array}$$

(3) $$\begin{array}{c} i_{t}=\sigma \left(U_{i}\left[h_{t-1},w_{t}\right]+b_{i}\right), \end{array}$$

(4) $$\begin{array}{c} {\bar{c}}_{t}=\sigma \left(U_{c}\left[h_{t-1},w_{t}\right]+b_{c}\right), \end{array}$$

(5) $$\begin{array}{c} c_{t}=f_{t}*c_{t-1}+i_{t}*{\bar{c}}_{t}, \end{array}$$

(6) $$\begin{array}{c} o_{t}=\sigma \left(U_{o}\left[h_{t-1},w_{t}\right]+b_{o}\right), \end{array}$$

(7) $$\begin{array}{c} h_{t}=o_{t}*\;\tan h\left(c_{t}\right), \end{array}$$

where *σ* is the logistic regression function; *U* denotes the matrix multiplication operation; *b* is the function bias term; tanh is the activation function; and *h*_*t*_ denotes the state of the memory cell.

Firstly, the sentence vector is generated by Bi LSTM; then the text vector *W* is generated by one layer of Bi LSTM, and then the text vector *W* and the domain knowledge topic vector *T* or the text topic vector *V* are sequentially stitched together. A text may contain more than one domain knowledge, corresponding to more than one domain knowledge topic vector *T*_*i*_ , and the method of generating the domain knowledge topic vector *T* is shown in equation (8). The vector order stitching method is shown in equation (9). This study expects that a more accurate representation of medical text vectors can be obtained than using text vectors alone, and it can be used to improve the text semantic similarity calculation.

(8) $$\begin{array}{c} T=\frac{1}{m}\sum_{1}^{m}T_{i}, \end{array}$$

(9) $$\begin{array}{c} G_{w}\left(D\right)=\left\{W,T\right\},G_{w}\left(D\right)=\left\{W,V\right\}. \end{array}$$

The Siamese Network framework input information is *E*_*w*_ and the labels *y* between the texts. This study calculates the distance between vectors *G*_*w*_ (*D*_1_) and *G*_*w*_ (*D*_2_) by the cosine similarity method *E*_*w*_. The text labels *y* are calculated using the BMA [13] (Best Match Average) method. This method mainly uses the domain knowledge information obtained from the full text and the domain knowledge topic vector obtained from the TWE model. The text labels are calculated as shown in Figure 6.

RETRACTED

As shown in Figure 6, assuming that there are two texts, *D*_1_ and *D*_2_, the domain knowledge extracted by the mark in *D*_1_ is (*A*_1_, *A*_2_, *A*_3_,…, *A*_*m*_) and the domain knowledge extracted by the mark in *D*_2_ is (*B*_1_, *B*_2_, *B*_3_,…, *B*_*n*_). According to Table 1, the subject distribution and vector representation of domain knowledge corresponding to each domain knowledge are obtained. Calculate the label *y* between texts *D*_1_ and *D*_2_ by the BMA method, as shown in formula (10):

(10) $$\begin{array}{c} y\left(D_{1},D_{2}\right)=\frac{1}{2}\left(\frac{1}{m}\sum_{A_{m}\in D_{1}}\max_{B_{n}\in D_{2}}\cos\left(T_{A_{m}},T_{B_{n}}\right)+\right.\left.\frac{1}{n}\sum_{B_{n}\in D_{2}}\max_{A_{m}\in D_{1}}\cos\left(T_{B_{n}},T_{A_{m}}\right)\right). \end{array}$$

To further improve the prediction performance of this study, the above annotation method is compared with the text topic-based annotation method, assuming that the text topics of the two articles are *v*_1_ and *v*_2_, and the text topic-based label *y* is calculated by cos(*v*_1_, *v*_2_). After selecting the best annotation method, the Siamese Network is used to learn the similarity measure between the two text vectors, which is validated by test set data and the similarity matrix between the texts is obtained for clustering analysis.

The loss function of the Siamese Network model is shown in equation (11):

(11) $$\begin{array}{c} L_{w}=\frac{1}{4}\left(1-E_{w}^{2}\right)y+\left(1-y\right)E_{w}^{2}. \end{array}$$

RETRACTED

## 4. Case Study

### 4.1. Source

Patients with urinary infections who had no indwelling catheters were included. According to the “Diagnosis and Treatment of Urinary Infections Chinese Experts' Common Knowledge” (2015 Edition) [6], the diagnostic criteria for asymptomatic bacteriuria, also known as asymptomatic urinary infection, in which a certain amount of bacteria is isolated from the urine specimen without any signs or symptoms of urinary infection in the patient, are a urine culture bacterial colony count ≥105 CFU/ml for asymptomatic female patients; 1 strain of bacteria colony count ≥103 CFU/ml for clean urine specimens cultured from male patients. Patients with urinary infections who did not meet the criteria for asymptomatic bacteriuria were included in the symptomatic urinary infection group.

### 4.2. Results

There was no statistically significant difference between the two groups in terms of age and gender. See Table 1.

The two groups of patients were mainly distributed in geriatric-related departments, with 21 cases in geriatric neurology accounting for 24.42% and 8 cases accounting for 18.18%, and 13 cases in geriatric cardiovascular department accounting for 15.12% and 10 cases accounting for 22.73%, respectively. See Table 2.

The antibacterial drug use rate was 94.19% (81/86) in the symptomatic urinary infection group than 77.27% (34/44) in the asymptomatic bacteriuria group, with a statistically significant difference (*χ*2 = 8.158, *P*=0.004); the duration of antibacterial drug use was 10.5 (6, 17.25) *d* more in the symptomatic urinary infection group than in the asymptomatic bacteriuria group (5 (1, 10) *d*), with a statistically significant difference (*Z* = −3.889, *P* < 0.001).

To further evaluate the diagnostic value of urinary leukocyte count in differentiating symptomatic urinary infection from asymptomatic bacteriuria, the ROC curves of urinary leukocytes in the two groups were plotted, and the area under the curve was 0.767 (95% CI: 0.666–0.869), and the cut-off value of urinary leukocytes was 231.90, with a sensitivity of 80.00% and specificity of 67.60%. The area under the curve of serum PCT in both groups was 0.739 (95% CI: 0.548–0.930), and the cut-off value of serum PCT was 0.0405, with a sensitivity of 100.00% and specificity of 57.10%. The urinary leukocyte and serum calcitoninogen ROC curves are shown in Figure 7.

With age, the systemic and local immune function of the elderly gradually declines, and the mucosa of the urinary tract and the bladder and other organs become atrophied and thin, resulting in reduced defense functions and susceptibility to infection; especially, elderly inpatients often have one or more chronic underlying diseases such as hypertension, diabetes, tumors, etc., and are at high risk for urinary tract infections. Urinary tract infections are usually differentiated into symptomatic urinary infections and asymptomatic bacteriuria according to the presence or absence of urinary irritation symptoms such as urinary frequency, urinary urgency, and urinary pain; there are essential differences in their anti-infective treatment modalities, except for the differences in clinical manifestations. Studies have confirmed [8] that the probability of asymptomatic bacteriuria in elderly women hospitalized in long-term care facilities is as high as 25% to 50%, and the probability of asymptomatic bacteriuria in elderly men is as high as 15% to 40%, as shown in Figure 8 for the analysis of different urinary tracts.

RETRACTED

Geriatric urinary infection patient units are mainly distributed in geriatric-related clinical departments, and patients are mostly hospitalized for a long time. The risk of urinary infection is much higher than that of geriatric patients in other non-geriatric departments, and clinical work should pay special attention to the risk of urinary infection in geriatric patients who are hospitalized for a long time. It is worth noting that elderly urological patients have a certain probability in asymptomatic bacteriuria, suggesting that surgical operations for urological diseases may increase the incidence of bacteriuria. The results of this study showed that the pathogenic bacteria were predominantly Gram-negative, with *Escherichia coli* predominating, which is consistent with the report [9] and similar to the distribution of pathogens in the whole population [10, 11]. In this study, after removing patients with the above indications for antimicrobial drug use, it was found that the rate of antimicrobial drug use in the asymptomatic bacteriuria group was as high as 77.27%, indicating that 77.27% of the use was unreasonable. The abuse of antimicrobial drugs not only cannot improve the chronic genitourinary symptoms of patients, but also increases the probability of double infection and increase adverse drug reactions, as shown in Figure 9 for different clustering effects.

## 5. Conclusions

In recent years, the incidence of cardiovascular diseases has increased as the number of elderly people in China has increased. The cardiology department is the main place to admit patients with cardiovascular diseases, which are characterized by long durations of illness, high age, low immune status, and many complications, and some patients need to perform invasive operations, which are very likely to induce nosocomial infections. The TWE model was used to represent word vectors and topic vectors in the study of urinary infections in elderly inpatients, and the similarity was calculated based on the Siamese Network framework combining text and domain knowledge topics.

RETRACTED

## Figures and Tables

**Figure 1:** Research framework.

**Figure 2:** Number of medical entity markers.

**Figure 3:** Statistical distribution of the number of genetic markers.

**Figure 4:** TWE model framework.

**Figure 5:** BiLSTM Siamese network framework.

**Figure 6:** Text label calculation method.

**Figure 7:** Urinary leukocytes and serum calcitoninogen ROC curves.

**Figure 8:** Analysis of different urinary tracts.

**Figure 9:** Different clustering effects.

**Table 1:** Clinical data of the two groups of patients.

Clinical data	Symptomatic urinary tract infection group (*n* = 86)	Asymptomatic bacteriuria group (*n* = 44)	Statistic	*P* value

0.136Gender (cases)	Male	49	19	2.22
	Female	37	25	

Age (years)	81.38 ± 10.75	80.16 ± 10.39	0.391	0.697

**Table 2:** Composition ratio of the distribution of infected departments in the two groups of patients.

Department	Symptomatic urinary tract infection group (*n* = 6)		Asymptomatic bacteriuria group (*n* = 44)	
	Number of cases	Composition ratio (%)	Number of cases	Composition ratio (%)

Geriatric neurology	21	24.42	8	18.18
Geriatric cardiovascular department	13	15.12	10	22.73
Geriatric nephrology	8	9.3	0	0
Geriatric respiratory department	7	8.14	3	6.82
Geriatric endocrinology department	5	5.81	0	0
Geriatric gastroenterology	0	0	4	9.09
Urology surgery	0	0	3	6.82
Other	32	37.21	16	36.36

## Data Availability

The data underlying the results presented in the study are available within the manuscript.
